# Effect of Social Beliefs on Consumption of Dairy Products and Its Predicting Factors Based on the Transtheoretical Model: A Population-Based Study

**DOI:** 10.1155/2023/5490068

**Published:** 2023-01-27

**Authors:** Veda Vakili, Kourosh Vakili, Mohammad Zamiri Bidari, Adele Azarshab, Mohammad Moein Vakilzadeh, Kiyoumars Kazempour

**Affiliations:** ^1^Department of Community Medicine and Public Health, Faculty of Medicine, Mashhad University of Medical Sciences, Mashhad, Iran; ^2^Faculty of Medicine, Mashhad University of Medical Sciences, Mashhad, Iran; ^3^Student Research Committee, Faculty of Medicine, Mashhad University of Medical Sciences, Mashhad, Iran

## Abstract

**Background:**

Social beliefs on the consumption of dairy products are associated with health conditions, and the aim of this study is to investigate associated factors with the rate of dairy product intake, in accordance with social health-related beliefs and the elements predicting dairy consumption, based on the transtheoretical Model (TTM).

**Methods:**

981 subjects (chosen from Mashhad citizens, Iran) were surveyed in random public places in 2014, using demographic surveys and questionnaires based on TTM and advantage/disadvantage by trained interviewers.

**Results:**

981 Subjects with a mean age of 30.39 ± 14.83 were surveyed in dairy nonconsumer and dairy consumer groups. There was a significant relationship between dairy consumption and gender (*P* < 0.001). Factors such as age, educational level, job status, and opium addiction were found to be significantly associated with dairy consumption status. Young and female subjects consume more dairy products than their older and male counterparts, respectively. People with a diploma degree and lower levels of education consumed substantially more dairy products than their educated equals. Unemployed participants consumed considerably more dairy products than their fellow employed participants. Opium-addicted subjects were more likely to avoid dairy products.

**Conclusions:**

Despite the general belief of dairy consumption being beneficial, subjects in the precontemplation stage as nonconsumers described dairy products as of poor taste having low diversity in markets. Also, among the reasons, dairies' short shelf-life and behaviours under the influence of society and family were the mains. The termination stage's subjects as consumers consumed dairy products mostly for losing weight.

## 1. Introduction

### 1.1. Background

Dairy products, including milk, are considered as rich nutrients. Despite their low-level calories, these products supply the elements required for the normal function of the organs [1–3], such as water, fat, necessary proteins, calcium, phosphorus, magnesium, potassium, zinc, selenium, and group of vitamins (A, E, K, B2, B5, and B12). As a preventive factor, these products lower the risk of diabetes, stroke, hypertension [4], bone fracture [5], cardiovascular diseases, and obesity [6]. According to the annual reports of the International Dairy Federation (IDF), the average global consumption of milk has risen gradually in the last decade (from 101.4 kg/capita/year in 2005 to 113 kg/capita/year in 2017) [7, 8]. Due to the latest reports of the Food and Agriculture Organization (FAO), low-fat and whole milk consumption in Iran is about 64.38 kg/capita/year [9], which is far lower than the global average.

Demographic and socioeconomic factors, such as price, availability, awareness, and convenience could affect dietary behavior [10]. Although, dairy industry in Iran is advance and also, During 1996–2001, dairy products involved just 2.5 percent of total Iranian family expenditure [11] but recently due to economic sanctions the dairy price increased as the family income decrease . In addition to, poor awareness of food values among people and lack of promotions of companies in Iranian society could lead to low dairy consumption [12]. In addition, if dairy products are not prepared under hygienic conditions, then it will lead to infection disease [13].

As the consumption of dairy products in Iran is lower than the world average, it is necessary to find predictors and related factors associated with this issue. Unlike Iran, there is promising evidence on attraction factors for dairy consumption [14].

The transtheoretical model (TTM) is an intentional method emerged from comparative analyses of approximately 300 psychotherapy theories [15]. This model is used for categorizing people into different stages towards specific health behaviors [16] and developing correct behaviors in each person individually according to his/her conditions [17].

According to controversies and lack of efficient studies on dairy products consumption, we decided to assess the related factors of dairy consumption and beliefs associated with the population's behavioral conditions based on TTM in Mashhad, Iran.

## 2. Methods

### 2.1. Study Design, Participants, and Data Collection

In 2014, 981 people were surveyed in our cross-sectional study in order to assess the local population's dairy product consumption and its predictors in Mashhad (second largest city of the country), Iran [18]. The multistage selection method was administered to select the participants. At the first step, we made a list of public sites such as parking lots, banks, hospitals, and universities belonging to municipal categorizations and urban maps all around the city; then, we assigned numbers to each site, and after that, we selected random numbers from the list. Then, at the second step, in each place, subjects were chosen by the random convenience method and interviewed by a trained interviewer. The criteria for selecting the subjects were literacy, being socially active, consent to participate in this study, and citizenship of Mashhad. Subjects consuming more than 3 units of dairy products were defined as consumers. Each unit of dairy food was defined as a glass of milk, a cup of yogurt, a cup of curd, a glass of ice cream, a matchbox of cheese or two glasses of “dough,” and a local salty beverage similar to soured milk. All the measures were drawn from the previous studies [19, 20].

### 2.2. Questionnaires

We designed a questionnaire consisting of two main sections. In the first section, due to the 6 stages of TTM, 6 yes/no questions were designed. Someone in the precontemplation stage had no tendency to consume dairy products within the last 6 months. In addition, subjects in the contemplation stage have not yet consumed dairy products but are planning to consume them in the following 6 months. Furthermore, participants in the preparation stage have taken some measures to modify their lifestyle and are planning to start dairy consumption within the next month. Participants starting dairy consumption in the last 6 months were classified in the action stage. The maintenance stage comprised people beginning consumption for 6 months or more. Finally, subjects in the termination stage do not have any intention to return to their previous unhealthy habits. The second section consisted of questions evaluating the subjects' beliefs on the advantages, disadvantages, and barriers to consuming recommended dairy products on a 5-point Likert scale. Validating the questionnaire was performed with expert council which included 6 experienced researchers [Table 1]. The internal consistency for total and subscales was calculated by Cronbach's alpha coefficient, and reliability between the test and retest was performed using the intraclass correlation coefficient (ICC). The total ICC was 0.90, and Cronbach's alpha was 0.65–0.74. We also added a sociodemographic checklist including age, gender, height, weight, job status, family income, educational level, marital status, household size, and exercise habits.

### 2.3. Ethics

Interviewers informed all people participating in this study of the aim of the research and ensured them of the confidentiality of their personal data. After oral consent, interviewers filled the questionnaire during a face-to-face conversation. The study was approved by the Ethics Committee of the Mashhad University of Medical Sciences (ethical approval code: 930054).

### 2.4. Statistical Analysis

The 16th version of the SPSS software (SPSS Inc., Chicago, Illinois, USA) was used for all statistical analyses. Data normalizations were checked by the Kolmogorov–Smirnov test. The chi-square test was used to examine the significance between categorical data. The Mann–Whitney test was applied for nonparametric data analyses. In order to eliminate the effects of confounding variables, logistic regression analysis was used in assessing pros/cons of items among the subjects of precontemplation and termination stages. All tests were 2-tailed, and probability values below 0.05 were deemed significant.

## 3. Results

### 3.1. Sociodemographic Characteristics

Table 2 depicts the sociodemographic characteristics of study participants. 981 people between 10 and 85 years randomly participated in our cross-sectional study. The mean age was 30.39 ± 14.83 (separately 34.61 ± 14.90 for males and 25.86 ± 13.28 for female participants). The study included 506 (51.58%) male subjects and 475 (48.41%) female subjects. 453 (46.17%) subjects were married, and 42.40% of them were employed. The participants' median BMI was 25.2 (22.5–27.6) and 22.1 (19.3–25.2) for men and women, respectively.

### 3.2. Patterns of Dairy Food Intake

In descending order for males, the ratio of consumption of yogurt, milk, cream, ice cream, cheese, and curd to total dairy consumption was 37.1%, 23.8%, 16.8%, 13.8%, 7%, and 1.6%, respectively. In addition, the previous pattern for women indicates that the ratio of consumption of yogurt, milk, cream, cheese, ice cream, and curd to total dairy consumption was 39.7%, 22.2%, 17.7%, 10.4%, 8.7%, and 1.3%, respectively.

### 3.3. Dairy Consumption Status

The transtheoretical Model for dairy product consumption indicated that the largest groups of men and women were at the termination stage. Moreover, the results demonstrated that in every 4 female, about 3 subjects (70.00%) consumed dairy products, whereas in males, some two thirds (61.06%) of the subjects consumed dairy products (Table 3).

### 3.4. Comparison between Dairy Consumers versus Nonconsumers

As discussed before, the first three stages (precontemplation, contemplation, and preparing) and the second three stages (action, maintenance, and termination) were categorized into dairy nonconsumer and dairy consumer groups, respectively. As shown in Table 4, the chi-square test showed a significant relationship between dairy consumption and gender (*P* < 0.001). Furthermore, we found factors such as age, educational level, job status, and opium addiction to be significantly associated with dairy consumption status. Young and female subjects consume more dairy products than their older and male counterparts, respectively. People with a diploma degree and lower levels of education consumed substantially more dairy products than their educated equals. Unemployed participants consumed considerably more dairy products than their fellow employed participants. Last but not least, opium-addicted subjects were more likely to avoid dairy products. No meaningful relationship was found between the subjects' marital status, family size, monthly income, and BMI in the consumer and nonconsumer groups (Table 4).

### 3.5. Subjects' Beliefs of Dairy Foods

Overall, our participants agreed with the benefits of consuming dairy products for their health. They also firmly believed in the consumption of dairy foods as a beneficial substitute for unhealthy diets. The most important factors leading to the lack of motivation were, from highest to lowest, the presence of preservatives in dairy products, limited sustainability, and high prices. Table 1 indicates the mean scores given by people for each advantage/disadvantage.

The multiple regression test was used to recognize most related beliefs in precontemplation and termination stages. So, we defined two extremes of consuming stages precontemplation and termination as outcome and participants believes as predictors.

As shown in Table 5, in the precontemplation stage, 6 items and their related beliefs are significantly associated with participants. Also, the benefits of consuming dairy products for general health and weight loss persuaded several subjects to take dairy products permanently in the termination stage.

## 4. Discussion

Milk and dairy products contain various necessary nutrients, such as calcium, phosphorus, magnesium, zinc, vitamins [21], and proteins, which are important for immunity, prevention of tumour development, and iron absorption. A recent study on the Iranian society has demonstrated that the consumption of skimmed milk as a common food has decreased considerably, from 65.39 kg/capita/year in 2007 to 46.69 kg/capita/year in 2013 [9].

We aimed to evaluate the factors affecting dairy consumption and assess social beliefs of citizens of the second biggest city in Iran about dairy products.

The participants' mean age was 30.39 ± 14.83, close to the Iranian population's mean age (31.10 years) which was unofficially declared by the Statistical Centre of Iran in 2016, indicating that in terms of age, this study could be a proper sample of Iranian people. Among participants, males are 3 times more employed than females, due to patriarchal circumstances in Iran. In addition, more than a half of male subjects have academic degree, even though 38.73% are graduated from college. Leaving college before graduation were because of males' tendency to acquire more comfortable, professional, and high-income jobs and form sustainable families in financial, behavioural, and social perspectives.

In a recent study on 56233 people with an age of 50 years and over, among 16 countries of Europe, confirms our results that women's higher knowledge about advantages of dairy products for health could lead to more dairy consumption [22]. In our study, females are significantly more motivated to consume dairy products than males, and overall, their percentage in the consumer group is higher than males. A study conducted by Green et al. found no significant relationship between gender and dairy consumption, even though they found a specific relationship between gender and milk consumption [23]. Mirmiran et al. indicated that among 462 subjects of 16 years and over, men consume significantly more dairy products than women [24]. Other studies based on children and adolescents demonstrated similar results to those reported by Larson et al. [25, 26]. We believe that the subjects' number, age range, and social conditions are responsible for these controversies.

Our results, similar to those of the study by Gopinath et al., imply an indirect relationship between subjects' age and dairy consumption [26]. According to educational level, in our study, subjects with diplomas and lower degrees were more likely to consume dairy foods. Among the Iranian populace, people of higher education, due to their higher ages, deal more difficulties in their daily lives and spend a lot of time in working environments. Thus, they cannot pay enough attention to their lifestyles and adjust them correctly.

In this study, opium-addicted people significantly utilize lower dairy foods than nonabusers. Despite the low percentage of addicted subjects in this study, this outcome confirms previous results that unhealthy behaviors are associated with a clustering pattern, performed in another Iranian metropolis, Shiraz, Iran [27].

Our study found no significant relationship between the BMI and dairy consumption. Similarly, in the prospective cohort study by Gopinath et al., the participants' (school children) BMI was not significantly related to high dairy consumption during 5 years of subjects' adolescence [26]. In contrast to our results, a cross-sectional research study by Mirmiran et al. showed an indirect moderate correlation (*r* = −.36, *P* value<0.05) between dairy servings and BMI [24]. Furthermore, a prospective cohort study found a significant inverse association between primary school children's BMI and frequency of dairy consumption. In this topic, our study subjects' BMI was self-reported, and due to the differences between study designs and subjects' age, the results could have also varied.

For evaluating the behavioral conditions of Mashhad citizens, we used multiple regression analysis, a very general system in the field of behavior assessment [28]. Due to the subjects scoring each item, we used multiple regression tests to analyse data in order to find significant pros and cons of dairy product consumption. According to the results of this test, even though nonconsumer subjects without the intention of consuming dairy foods in the precontemplation stage believed in benefits of dairy products for their health and diet, they argued that common and available dairy products are of poor taste and have low diversity in markets. Also, they believe that dairy products' relatively short expiration date could be an issue. Last but not least, peer pressure and social and family impacts in the precontemplation stage are proven as important factors leading to an unhealthy diet. We found that their knowledge of dairy products' health advantages, such as efficacy to weight control, was significant factors for the participants consuming dairy products and satisfied with their dairy diet habit..

This study was administered on a large population randomly selected from public places. Thus, it could be highly good representative of our study population. Furthermore, we used the multiple regression test as a very general and useful test for analysing people's behavioral situations. To the best of our knowledge, this is the first pro/con study performed in the field of dairy consumption which was analysed by the logistic regression test.

The most important limitation of the current study was its study design since we did not follow up the subjects participating in this research. Moreover, all data collected by written surveys were self-reported, and hence, their measurable characteristics such as height and weight were not verified by using standard instruments and methods.

As mentioned before, we found no previous studies assessing the effects of population beliefs on diet behaviors in consuming dairy foods. Therefore, we recommend future studies to evaluate this issue in order to find out factors alienating people from dairy products and solve them by purposeful advertisements and conscious decisions in dairy industries to convince people to include dairy products in their diet. In addition, we advise researchers to design large longitudinal studies determining predictors of dairy consumption, particularly due to controversies between previous researches.

## 5. Conclusions

This study demonstrated that young, female, unmarried, and unemployed people were significantly more dispersed in consumer groups and that opium-addicted subjects were more in the nonconsumer group. Moreover, despite the general belief of dairy consumption being beneficial, subjects in the pre-contemplation stage, as non-consumer, described dairy products as of poor taste and diversity in the markets. Also, among the reasons, dairies' short shelf-life and behaviours under the influence of society and family were the mains. The termination stage's subjects as consumers consumed dairy products mostly for losing weight.

## Figures and Tables

**Table 1:** People's scores depending on their agreement with beliefs mentioned in the questionnaire.

Advantage questions	Scores/5 Mean ± SD
1. Consuming dairy products is good for your body	4.19 ± 0.92
2. Eating dairy products can help prevent diseases	4.19 ± 0.89
3. Dairy products could be a good alternative for unhealthy food products	3.99 ± 1.05
4. Eating dairy products makes human beings feel happy and joyful	3.68 ± 1.17
5. Dairy products cause diversity in diet	3.66 ± 1.09
6. Advertisements are effective in the people consumption rate	3.64 ± 1.30
7. My religion recommends us to consume dairy products	3.63 ± 1.31
8. Consuming dairy foods can help people lose their weight	3.55 ± 1.27
9. Other people eat dairy products too	3.11 ± 1.39

Disadvantage questions	

1. I Worry about the chemicals used in dairy products	4.13 ± 1.20
2. Dairy products soon become damaged and their use time is limited	3.58 ± 1.26
3. Dairy foods are expensive	3.56 ± 1.41
4. Advertisements on dairy intake are not enough	3.48 ± 1.39
5. Dairy consumption is not common in family and society	3.42 ± 1.34
6. Most dairy products are tasteless or taste bad	3.30 ± 1.36
7. Dairy diversity in the markets is low	3.22 ± 1.31
8. It is hard to find a delicious dairy product	3.18 ± 1.31

SD: standard deviation.

**Table 2:** Demographic and socioeconomic characteristics of the study sample (*n* = 981).

Participants characteristics		Male (*n* = 506) *N* (%) or mean (IQR)	Female (*n* = 475) *N* (%) or mean (IQR)
Educational level	High school and lower	208 (41.10)	275 (57.89)
	Completed college	297 (58.69)	184 (38.73)
	Missing	1 (0.19)	16 (3.36)

Job status	Employee	312 (62.20)	104 (22.12)
	Unemployed	190 (37.80)	371 (77.87)
	Missing	4 (0.79)	0 (0.00)

Abuse (alcohol or cigarette)	Yes	84 (16.60)	9 (1.89)
	No	422 (83.39)	466 (98.10)

Opium addiction	Yes	17 (3.35)	1 (0.21)
	No	489 (96.64)	474 (99.78)

Recommended physical activity	Yes	297 (58.69)	250 (52.63)
	No	209 (41.30)	225 (47.36)

Income (dollars per month)		433 (233–1000)	333 (166–666)

Body mass index (Kg/m^2^)		25.2 (22.5–27.6)	22.1 (19.3–25.2)

IQR: interquartile range.

**Table 3:** Participant frequency in each stage of TTM based on gender and dairy consumption.

Change stages		Male (*n* = 506) *N* (%) or mean (IQR)	Female (*n* = 475) *N* (%) or mean (IQR)
Nonconsumer (*n* = 280)	Precontemplation	59 (11.66)	34 (7.15)
	Contemplation	67 (13.24)	39 (8.21)
	Preparing	43 (8.49)	38 (8.00)
	Total	169 (33.39)	111 (23.31)

Consumer (*n* = 642)	Action	69 (13.63)	39 (8.21)
	Maintenance	59 (11.66)	95 (20.00)
	Termination	181 (35.77)	199 (41.89)
	Total	309 (61.06)	333 (70.10)

Total missing (*n* = 59)		28 (5.53)	31 (6.52)

IQR: interquartile range.

**Table 4:** Comparison of demographic characteristics and dairy product consumption between consumer and nonconsumer groups.

Demographic characteristics		Nonconsumer (*N* = 280) *N* (%) or mean (IQR)	Consumer (*N* = 642) *N* (%) or mean (IQR)	*P* Value
Gender	Male	169 (35.35)	309 (64.64)	<0.001^a^
	Female	111 (25.00)	333 (75.00)	

Age (Years)		28 (20–39)	26 (19–40)	0.030^b^

Household size (no.)		4 (3–5)	4 (3–5)	0.450^b^

Marital status (married)		142 (50.71)	311 (48.44)	0.230^a^

Educational level (completed high school and lower)		116 (41.42)	336 (52.33)	0.004^a^

Job (employed)		135 (48.21)	263 (40.96)	0.040^a^

Opium addiction (yes)		13 (4.64)	5 (0.77)	<0.001^a^

Income (dollars per month)		400 (220–1000)	333 (216–833)	0.470^b^

Body mass index (Kg/m^2^)		24.20 (21.40–26.60)	23.80 (20.70–26.80)	0.650^b^

^a^Chi-square test. ^b^Mann–Whitney test. IQR: interquartile range.

**Table 5:** Significant advantage/disadvantage questions for subjects classified in the precontemplation stage and the termination stage.

Change stage	OR	*P* value^a^
Pre-contemplation		
Eating dairy products is good for your body	3.448	<0.001
Dairy products cause diversity in diet	1.845	0.022
It is hard to find delicious dairy products	1.996	0.003
Dairy diversity in the markets is low	0.654	0.035
Dairy products will go bad early and their shelf-life is limited	1.875	0.003
Dairy consumption is not common in family and society	0.412	<0.001
Termination		
Eating dairy products is good for your body	0.460	<0.001
Consuming dairy foods can help people with an intention to lose weight	1.417	0.006

^a^Logistic regression test. OR: odds ratio.

## Data Availability

Data are available on reasonable request from the corresponding author.
